This article has been retracted.

# Preventive Effect Observation of Dapagliflozin on Middle and Later Ventricular Remodeling in Patients with Acute ST Segment Elevation Anterior Wall Myocardial Infarction: A Single-Center, Retrospective Cohort Study

**DOI:** 10.1155/2022/3955914

**Published:** 2022-04-15

**Authors:** Zeyan Liu, Lijun Liu, Hao Zhang, Yang Jiang, Hengtong Wang

**Affiliations:** ^1^Department of Emergency Internal Medicine, The Second Hospital of Anhui Medical University, Anhui, Hefei 230000, China; ^2^Department of Emergency and Critical Medicine, The Second Affiliated Hospital of Soochow University, Jiangsu, Suzhou 215000, China; ^3^Department of Emergency Internal Medicine, The Fourth Hospital of Anhui Medical University, Anhui, Hefei 230000, China

## Abstract

*Objective*: This study aimed to observe the effect of dapagliflozin on left ventricular ejection function (LVEF) and left ventricular end-diastolic volume (LVEDV) in patients with acute anesthesia ST segment elevation myocardial infarction (ASTEMI) and explore the effect of prophylactic treatment on ventricular remodeling (VR). *Methods*. A retrospective cohort design was employed to collect 188 patients with anterior wall STEMI who received emergency percutaneous coronary intervention (PCI). The patients were divided into dapagliflozin group and control group. The baseline data, the results of echocardiography at 6 months and on admission, and the proportion of VR were compared between the two groups. Echocardiography followed up for the two groups for 6 months after PCI and VR (LVEDV increased ≥20%) were considered the main clinical outcomes. Single-factor and multifactor logistic regression was conducted to explore the preventive effect of dapagliflozin on VR in patients with anterior wall STEMI. *Results*. There were significant differences in gender, history of diabetes, glycosylated hemoglobin (Hb1AC), admission LVEF, Killip grade of heart failure, and brain natriuretic peptide (BNP) between the dapagliflozin group and the control group regarding the baseline data. Compared with the results of echocardiography at admission and 6 months, the decrease in LVEDV and the increase of LVEF at 6 months in the dapagliflozin group were significantly higher than those in the control group. During the follow-up of 6 months, the VR rate in the dapagliflozin group was significantly lower than that in the control group. Multifactor logistic regression analysis suggested that the risk of VR was reduced by taking dapagliflozin after the adjustment of the confounding factors. Additionally, the combined use of dapagliflozin, ACEI/ARB, and *β*-block can further reduce the risk. *Conclusion*. Regular taking of dapagliflozin has a positive effect on the improvement of middle and LVEF and left ventricular volume enlargement in patients with anterior wall STEMI, as well as the prevention of the occurrence of VR.

## 1. Introduction

Acute ST segment elevation myocardial infarction (STEMI) is a cardiovascular disease severely influencing the national survival time and quality [1]. The establishment of a chest pain center and the popularization of emergency percutaneous coronary intervention (PCI) significantly reduce mortality in the acute phase of STEMI. However, the mortality rate in the middle and later stages of STEMI is still on the rise, according to the epidemiological investigation [2]. Ventricular remodeling is the main pathological cardiac structural change leading to the decrease of cardiac ejection fraction in the middle and later stages of STEMI patients, as well as the main cause of mortality in the middle and later stages [3]. It is currently believed that acute ischemia is only the initiating factor of remodeling, and cardiomyocyte apoptosis, inflammation, and myocardial interstitial fibrosis caused by ischemia through various biological pathways are the direct causes of ventricular remodeling. Although the occluded vessels are opened in the time window, remodeling cannot be completely avoided [4]. Clinical treatment of ventricular remodeling after STEMI is mainly achieved by combined drugs, such as ACEI/ARB and *β*-block. Nevertheless, the clinical effect is not satisfactory. The statistics suggest that the incidence of ventricular remodeling in STEMI patients under combined therapy is still 25% and 30%. Dapagliflozin is an inhibitor of sodium-glucose cotransporter 2 (SGLT2i). Basic studies have demonstrated that SGLT2i can reduce left ventricular volume load, improve interstitial fibrosis, lower myocardial inflammation, promote cardiomyocyte energy metabolism, and weaken cardiomyocyte apoptosis. This is the theoretical basis for preventing ventricular remodeling after STEMI. The 2021 ESC Heart failure guidelines revealed that dapagliflozin can reduce the risk of hospitalization and cardiovascular death in patients with heart failure of reduced ejection fraction (HFrEF) w/o diabetes [5]. Compared with ejection fraction in the functional evaluation of heart failure after STEMI, ventricular remodeling focuses on structural evaluation, which is a description of the same disease state from different perspectives. Therefore, dapagliflozin may improve the middle and later cardiac ejection function and reduce the occurrence of ventricular remodeling in patients with STEMI. In this study, a retrospective cohort study was conducted to observe the preventive effect of dapagliflozin on ventricular remodeling after STEMI, so as to lay a theoretical foundation for clinical treatment strategies.

## 2. Materials and Methods

### 2.1. Study Design and Population

This study was a single-center, retrospective cohort study. Patients with STEMI in the anterior wall of the Chest Pain Center of the Second Hospital of Anhui Medical University from May 2020 to May 2021 were collected. This study was approved by the Ethics Committee of the Second Hospital of Anhui Medical University (PJ-YX2020-014 (F1)).

 
*Inclusion criteria:* (1) The diagnosis is in accordance with the fourth version of the STEMI global definition, and coronary angiography confirms that the left anterior descending is the anterior wall myocardial infarction of the target vessel; (2) the relevant clinical data is available from the chest pain center database and hospital medical record system; (3) if the time window of onset is less than 24 hours, the direct PCI treatment is performed with the time of D2W less than 90 min; (4) age: 45 to 75 years old.
 
*Exclusion criteria:* (1) combined with severe hepatic and renal function injury or other organ injuries; (2) complicated with malignant tumor; (3) combined with rheumatic immune disease; (4) they have valvular heart disease, Cor pulmonale, hypertensive heart disease, and cardiomyopathy at the same time; (5) the blood flow of the left anterior descending still did not reach Thrombolysis in myocardial infarction 3 (TIMI3) grade at the end of the operation; (6) there is a serious lack of medical records; (7) follow-up cannot be completed through coordination; (8) patients who have taken dapagliflozin to treat related diseases.

199 patients were enrolled through the inquiry of medical records and the inclusion and exclusion criteria. The patients were divided into two groups according to whether they took dapagliflozin or not after the PCI operation. In the dapagliflozin group, 13 cases were eliminated (7 cases were lost to follow-up, and 6 cases were discontinued to take dapagliflozin), and 82 cases remained. In the control group, 8 cases were eliminated (5 cases were lost to follow-up and 3 cases took dapagliflozin midway), and 96 cases remained.

### 2.2. Data Collection

The demographic data and clinical data (disease data, blood test data, coronary angiography data, and echocardiography data) of 2 groups during admission were collected based on the case data.

(1) Demographic data (three indicators): gender, age, body mass index (BMI); (2) disease-related data (ten indicators): history of smoking, history of hypertension, history of diabetes, time of onset, time from entrance to smooth passage of occluded blood vessel with a guidewire (D2W), whether ACEI/ARB (angiotensin-converting enzyme inhibitors/Angiotensin II receptor blockers) is taken, whether *β*-block is taken, admission Killip grade, complicated with atrial fibrillation, complicated with ventricular arrhythmia; (3) Echocardiography data (three indicators): left ventricular ejection function (LVEF) on admission, left ventricular end-diastolic volume (LVEDV) at admission, maximum velocity of the mitral valve at early diastole on admission; (4) Coronary angiography indicators (three indicators): SYNTAX score, number of diseased coronary vessels, grade of collateral circulation; (5) Blood test indicators (eleven indicators): uric acid, glycosylated hemoglobin, low-density lipoprotein, high-density lipoprotein, brain natriuretic peptide (BNP), troponin I (CnTI), creatinine, glutamic pyruvic transaminase, fibrinogen (FDP), neutrophil/lymphocyte (NLR), platelet count.

### 2.3. Follow-Up

The results of echocardiography 6 months after PCI operation in 2 groups were followed up. The increase in LVEDV of echocardiography ≥20% after 6 months compared to the period of admission was regarded as the standard of ventricular remodeling [6].

### 2.4. Statistical Analysis

The data was analyzed by SPSS 24.0 statistical software. The measurement data is expressed as mean ± standard deviation (SD). The counting data are statistically described by frequency and constituent ratio. The independent sample *t*-test and analysis of variance were performed for the measurement data that accorded with the normal distribution and meet the homogeneity of variance. Meanwhile, a *t*-test was adopted for those that did not satisfy the homogeneity of variance. Besides, *χ*^2^ test and Fisher's accurate test were conducted for the measurement data comparison. The difference between the prerepeated measurement data and the postrepeated measurement data was calculated. The differences between the two groups were compared using the Mann–Whiney *U* rank-sum test. Logistics analysis was performed to analyze the clinical outcome of patients. The Enter method was used first, followed by the Forward: LR method (inclusion: 0.05, exclusion: 0.1). *P* < 0.05 was considered statistically significant.

## 3. Results

### 3.1. Basic Information

The results in Table 1 suggested no differences in age, BMI, history of smoking, history of hypertension, onset time, D2W time, admission LVEDV, maximum velocity of the early diastolic mitral valve, ACEI/ARB taking, *β*-block taking, atrial fibrillation, malignant ventricular arrhythmia, number of diseased coronary vessels, SYNTAX score, collateral circulation, uric acid, low-density lipoprotein, high-density lipoprotein, creatinine, glutamic pyruvic transaminase, FDP, CnTI, and NLR between the two groups. The difference was not statistically significant (*P* > 0.05). The gender, history of diabetes, and the proportion of Killip grade were not completely the same between the two groups, with a statistically significant difference (*P* < 0.05). Additionally, the LVEF of admission in the control group was higher than that in the dapagliflozin group, and the Hb1AC and BNP in the dapagliflozin group were higher than those in the control group.

### 3.2. LVEDV and LVEF at Admission and 6 months after Admission in Both Groups

Table 2 indicated that the reduction of LVEDV 6 months after admission in the dapagliflozin group was significantly higher compared to the control group regarding the baseline, presenting a statistically significant difference (*P* < 0.01). The results demonstrated that the use of dapagliflozin for 6 months could significantly reduce the LVEDV; the increase in LVEF 6 months after admission in the dapagliflozin group was higher than that in the control group, with a statistically significant difference (*P* < 0.01). It suggested that the use of dapagliflozin for 6 months can significantly increase LVEF. The changing trend of LVEDV and LVEF in the two groups is illustrated in Figures 1 and 2.

### 3.3. Comparison of Clinical Outcomes between the Two Groups of Patients

In Table 3, the proportion of ventricular remodeling after 6 months in the dapagliflozin group was lower than that in the control group, exhibiting a statistically significant difference (*P* < 0.05). The results revealed that the probability of ventricular remodeling decreased after 6 months of use of dapagliflozin.

### 3.4. Single-Factor Analysis of Ventricular Remodeling

The clinical outcome (ventricular remodeling) of the patients was analyzed through logistics regression to explore the effects of taking dapagliflozin, taking ACEI/ARB, taking *β*-block, LVEDV, LVEF, BNP, NLR, Hb1AC, history of diabetes, uric acid, and CnTI on admission on the prognosis. The Enter method was used. The results in Table 4 suggested that dapagliflozin taking, ACEI/ARB taking, *β*-block taking, and admission LVEF were prognostic protective factors, and the difference is statistically significant (*P* < 0.05); CnTI, BNP, and NLR were prognostic risk factors of patients, and the difference is statistically significant (*P* < 0.05); left ventricular end-diastolic diameter, uric acid, diabetic history, and Hb1AC did not influence the prognosis of patients, and the difference was not statistically significant (*P* > 0.05).

### 3.5. Multifactor Analysis of the Effect of Dapagliflozin on Ventricular Remodeling

The prognosis of patients (ventricular remodeling) was analyzed by logistics regression, as well as the effect of taking dapagliflozin on the prognosis of patients. Before and after the adjustment of the confounding factors, the use of dapagliflozin was the protective factor of ventricular remodeling. The results in Table 5 suggest that the use of dapagliflozin can still benefit patients with myocardial infarction and reduce the risk of ventricular remodeling after myocardial infarction under the combined action of various clinical factors affecting ventricular remodeling.

### 3.6. Multifactor Analysis of the Effect of Combined Use of Three Drugs on Ventricular Remodeling

The clinical outcome (ventricular remodeling) of the patients was analyzed through logistics regression to reveal the effect of taking dapagliflozin + ACEL/ARB+ *β* receptor blocker on the prognosis of the patients. Before and after the adjustment of the confounding factors, the use of the three drugs was a protective factor for ventricular remodeling. The results in Table 6 reflect that the combination of dapagliflozin and ACEL/ARB+ *β* receptor blockers can reduce the risk of ventricular remodeling after myocardial infarction under the combined action of various clinical factors affecting ventricular remodeling. Moreover, the preventive effect is better than that of taking dapagliflozin alone.

## 4. Discussions

Ventricular remodeling is a major change in the rational structure of heart disease that leads to high mortality in patients with STEMI in the middle and later stages [7]. The left ventricle is the main power pump for cardiac ejection, with left bundle branches and a large number of Purkinje fibers distributed. The reconstructed left ventricle, as the main target of remodeling, has not only thinning of the ventricular wall and volume expansion, but also severe abnormalities in ejection function and cardiac electrical conduction function. The left anterior descending (LAD), as the most imperative blood supply to the left ventricular wall, is responsible for the blood supply to the myocardium and conduction bundles of the anterior wall, anterior septum, apex, and part of the lateral wall of the left ventricle. Therefore, LAD occlusion can result in severe left ventricular wall ischemia. From one perspective, it directly causes cardiomyocyte necrosis. From another perspective, ischemia, an initiating factor, leads to severe inflammation in the left ventricular necrotic area, surrounding injury area, and ischemic area through different biological pathways, such as the RASS pathway, TGF-*β*/Smad pathway, and STAT3 pathway. In addition to ischemic and hypoxic necrosis of cardiomyocytes [8], there is a large amount of apoptosis in noninfarcted areas [9], extensive myocardial interstitial fibrosis, and collagen deposition [10]. The above pathological changes not only cause left ventricular enlargement in morphology, but also seriously affect the physiological function of cardiomyocytes, such as excitation-contraction coupling, endoplasmic reticulum Ca2+ uptake and release, cross-bridge movement, mitochondrial ATP energy metabolism, and electrical signal transduction [11]. Clinical manifestations include the continuous decline of cardiac diastolic-systolic function, malignant ventricular arrhythmias, and even sudden death.

Dapagliflozin is a renal tubular sodium-glucose symporter inhibitor (SGLT2i). It is mainly used to reduce the reabsorption of urine glucose and then lower blood glucose by inhibiting renal tubular sodium-glucose symporter. Meanwhile, the osmotic diuretic effect is enhanced due to the decrease of glucose reabsorption in urine, contributing to reducing the cardiac volume load to a certain extent [12]. As a result, the left ventricular enlargement caused by the high load is weakened. In recent years, other mechanisms of the drug have been gradually discovered. Lee et al. [13] confirmed that dapagliflozin can inhibit TGF-*β* pathway and reduce the degree of myocardial interstitial fibrosis. Gager et al. [14] proposed that dapagliflozin can inhibit the production of peroxides (ROS) and reduce myocardial inflammation. Maejima et al. [15] discovered that dapagliflozin reduced cardiomyocyte apoptosis mediated by mitochondrial dysfunction through the improvement of mitochondrial energy metabolism and the regulation of mitochondrial Ca^2+^ homeostasis in the animal model of heart failure. Myocardial interstitial fibrosis, cardiomyocyte inflammation, and cardiomyocyte apoptosis constitute the main pathological basis of ventricular remodeling after STEMI. Therefore, there is a theoretical foundation for dapagliflozin to prevent ventricular remodeling after STEMI.

At present, dapagliflozin can reduce the incidence of Major Adverse Cardiovascular Events (MACE) and mortality in patients with HFrEF and can be used as a first-line drug for the treatment of heart failure in patients with diabetes or nondiabetes, according to the 2021 ESC Heart failure guidelines [5]. Regarding patients with anterior wall STEMI, severe heart failure in the acute phase often indicates an increase in the probability of ventricular remodeling in the middle and later stages. Qin et al. [16] demonstrated a correlation between acute heart failure and ventricular remodeling in STEMI. Turkieh et al. [17] further confirmed a positive linear correlation between BNP indicator and ventricular remodeling in patients with STEMI on admission. The cause of severe heart failure in the acute stage of STEMI is also the main factor in promoting ventricular remodeling in the middle and later stage, that is, myocardial necrosis directly caused by ischemia and inflammatory reaction, apoptosis, and interstitial fibrosis induced by ischemia as an initiating factor. As mentioned earlier, dapagliflozin has the pharmacological effect of interfering with the abovementioned pathological reaction. Besides, some researchers revealed that middle and later ventricular remodeling and decreased ejection fraction in patients with anterior wall STEMI describe heart failure from different angles (morphology and function). Therefore, the clinical effect of dapagliflozin in the treatment of heart failure could also be reflected in the prevention of ventricular remodeling in the middle and later stages of STEMI.

In this study, the baseline data included a total of 30 indicators, except for gender, and only 6 factors had statistical differences. Among them, ACEI/ARB and *β*-block are effective drugs to prevent ventricular remodeling. In this study, there is no difference in whether the two groups took these drugs, indicating that the interference of the above drugs on the outcome observation is excluded. Additionally, there was no difference in onset time and D2W time between the two groups. This reflected that the ischemic time and revascularization time were similar between the two groups, and there was no difference in the effect of ischemic injury between the two groups. Furthermore, the distribution of the two groups of baseline data is balanced and comparable. The different factors of baseline data are mainly divided into two categories: heart failure indicators (admission LVEF, BNP, heart failure Killip grade) and diabetes indicators (history of diabetes, glycosylated hemoglobin). Among them, LVEF in the dapagliflozin group was significantly lower than that in the control group on admission, while the Killip grade and BNP in the heart failure group were higher than those in the control group. In other words, many patients with acute heart failure after anterior wall STEMI were treated with dapagliflozin in this study. This is consistent with the recommended medication strategy of the latest ESC guidelines for heart failure. Meanwhile, there are more patients with a history of diabetes and higher glycosylated hemoglobin value in the dapagliflozin group, revealing that STEMI patients with diabetes were more likely to use dapagliflozin in this study owing to the hypoglycemic effect of dapagliflozin.

In this study, echocardiography suggested that the increase of LVEF in patients with anterior wall STEMI 6 months later was higher than that in the control group at the time of admission. Therefore, the left ventricular blood pumping function induced by STEMI was improved to some extent in patients with anterior wall STEMI who received standard treatment for 6 months, consistent with the clinical findings of Packer et al. [18]. Yurista et al. [19] confirmed in animal experiments that the above effects are associated with reducing the inflammatory injury of cardiomyocytes after STEMI, improving the decompensation of cardiac ejection function caused by high volume load, and weakening cardiomyocyte apoptosis outside the left ventricular necrotic area. Six months later, the decrease of left ventricular volume in the dapagliflozin group regarding the baseline was higher than that in the control group, implying that dapagliflozin not only improved cardiac function, but also had a certain effect on left ventricular pathological enlargement caused by anterior wall STEMI. After analysis of causes, it is discovered to be correlated with relieving left ventricular volume load, myocardial interstitial fibrosis, and collagen deposition caused by ischemia. Li et al. [20] presented that SGLT2i relieved ventricular pathological enlargement by improving the degree of myocardial interstitial fibrosis in rats with myocardial infarction. Dhingra et al. [21] also verified that dapagliflozin can improve the increase of ventricular volume in patients with STEMI in the middle and later stage through cardiac MRI verification at the clinical level.

This study is not aimed at patients with STEMI, though Gamaza-Chulián et al. [22] confirmed the protective effect of SGLT2i on ventricular remodeling through a prospective cohort study. In this study, the subjects were patients with anterior wall STEMI, which were more targeted. The simple correlation comparison of the clinical outcomes in the two groups during the follow-up of 6 months revealed that the rate of ventricular remodeling in the dapagliflozin group was lower than that in the control group. This reflects that the standardized treatment with dapagliflozin can reduce the occurrence of ventricular remodeling after STEMI to a certain extent and has a certain preventive effect.

Subsequently, further statistical analysis was performed in this study based on simple correlation analysis. Exposure factors (taking dapagliflozin) were included as the main observation factors; baseline difference factors and clinically confirmed factors affecting ventricular remodeling were selectively included as potential confounding factors. Ventricular remodeling was taken as the clinical outcome. The single-factor logistic regression analysis suggested that ACEI/ARB, *β*-block, admission LVEF, BNP, NLR, and CnTI were confounding factors. Then, the multifactor logistic regression analysis was conducted. It was revealed that taking dapagliflozin was the protective factor of ventricular remodeling before and after the adjustment of the confounding factors. Thus, taking dapagliflozin could still benefit patients with anterior wall STEMI and reduce the risk of ventricular remodeling in the middle and later stage in practical clinical application under the combined action of various factors affecting ventricular remodeling. According to the specific analysis of the related confounding factors, ACEI/ARB, *β*-block, and admission LVEF were protective factors, while BNP, NLR, and CnTI were risk factors. The lower the admission LVEF, and the higher the BNP, the more severe the acute heart failure, and the greater the risk of ventricular remodeling in the middle and later stage. NLR, as an evaluation indicator of inflammation, can reflect the degree of myocardial inflammation caused by acute ischemia. The higher the value, the higher the probability of remodeling of heart failure. Seropian et al. [7] revealed that severe inflammatory injury is an essential factor resulting in ventricular remodeling. CnTI is one of the intracellular contraction coupling proteins in cardiomyocytes. During STEMI, cardiomyocytes are ischemic-injured-necrotic, and a large amount of CnTI is released into the blood. The quantitative value of peripheral blood not only indicates the severity of the myocardial injury, but also has a positive correlation with the risk of ventricular remodeling. Fertin et al. [23] demonstrated that the increase of CnTI was independently related to the occurrence of ventricular remodeling. ACEI/ARB and *β*-block drugs, which are classic antiventricular remodeling drugs, acting by inhibiting the RASS system and sympathetic nervous system, respectively [24, 25]. Concerning pharmacological mechanism, dapagliflozin is different from ACEI/ARB and *β*-block in action targets. No relationship between dapagliflozin and the RASS system or sympathetic nervous system has been discovered in related studies.

Finally, logistic regression was conducted to analyze the effect of the combined use of SGLT2+ACEL/ARB+ *β*-block on ventricular remodeling in patients. After the interference of confounding factors was excluded, the combination of three drugs can further reduce the risk of ventricular remodeling in the middle and later stages of STEMI. According to the analysis of the reasons, the mechanism of action of dapagliflozin is different from that of ACEI/ARB and *β*-block. Besides, the analysis of the mechanism of action of dapagliflozin revealed that dapagliflozin can improve the state of acute heart failure, reduce myocardial inflammation, and weaken cardiomyocyte injury in patients with STEMI through non-RASS and nonsympathetic pathways, so as to produce the clinical effect of preventing ventricular remodeling. This is a powerful supplement to the existing clinical strategies for the prevention of ventricular remodeling after STEMI. Lee et al. [26] suggested that the STAT3 pathway may be the target pathway for SGLT2i to reduce the inflammatory response. Xie et al. [27] conducted an *in vitro* experiment, demonstrating that the AMPK/mTOR pathway is one of the key targets for SGLT2i to improve cardiomyocyte apoptosis. Tian et al. [28] validated that SGLT2i can alleviate myocardial interstitial fibrosis after STEMI by inhibiting the expression of the TGF-*β* pathway. Therefore, in clinical application, dapagliflozin in combination with ACEI/ARB and *β*-block can coordinate in many ways to improve the clinical prevention effect.

There are some limitations to this study as follows: (1) inadequate source of cases in the single-center study and lack of a good representative sample; (2) this study is an observational study, and the conclusions still need to be further validated by large-scale randomized controlled studies; (3) cardiac magnetic resonance is more accurate than cardiac ultrasound in measuring left ventricular diastolic volume (determining whether ventricular remodeling is present).

To sum up, dapagliflozin is a new first-line drug for the treatment of heart failure, and there is a theoretical foundation for it to prevent ventricular remodeling after STEMI. This study demonstrated that dapagliflozin can effectively improve left ventricular ejection function and left ventricular volume and prevent the occurrence of ventricular remodeling in the middle and later stages of STEMI. However, this study is a single-center observational study, with a small sample size and limited sample sources. The research conclusions still need to be further verified by multicenter prospective randomized controlled trials.

## Figures and Tables

**Figure 1:** Comparison of left ventricular end-diastolic volume (LVEDV) at baseline and after 6 months between the two groups of patients.

**Figure 2:** Comparison of left ventricular ejection function (LVEF) at baseline and after 6 months between the two groups of patients.

**Table 1:** Comparison of basic characteristic data between two groups of patients.

Variable	Control group (*n* = 96)	Dapagliflozin group (*n* = 82)	*t/χ* ^2^	*P*
*General information*				
Age	60.90 ± 13.11	59.89 ± 13.60	0.501	0.617

*Gender*				
Male	57(59.4)	30(36.6)	9.192	0.002
Female	39(40.6)	52(63.4)		

BMI (metrological expression)	23.68 ± 2.04	23.95 ± 2.06	−0.889	0.375
*BMI (count expression)*				
Normal	64(66.7)	52(63.4)	0.214	0.830
Overweight	32(33.3)	30(36.6)		

*History of smoking*				
No	64(66.7)	58(70.7)	0.339	0.560
Yes	32(33.3)	24(29.3)		

*History of diabetes*				
No	50(52.1)	27(32.9)	6.612	0.010
Yes	46(47.9)	55(67.1)		

*History of hypertension*				
No	50(52.1)	41(50.0)	0.077	0.782
Yes	46(47.9)	41(50.0)		
Onset time (h)	8.69 ± 3.37	8.98 ± 3.50	−0.558	0.578
D2W (min)	60.35 ± 15.06	59.09 ± 14.25	0.574	0.567

*Information for echocardiography*				
Left ventricular ejection fraction on admission	42.21 ± 7.66	38.99 ± 8.49	2.660	0.009
Left ventricular end-diastolic volume on admission	153.05 ± 13.54	164.00 ± 18.46	-0.946	0.346
Maximum velocity of the mitral valve in early diastole	0.48 ± 0.29	0.46 ± 0.30	0.477	0.634

*Information on drug use and complications*				
Taking ACEI/ARB				
No	16(16.7)	19(23.2)	1.184	0.276
Yes	80(83.3)	63(76.8)		
Taking *β*-block				
No	19(19.8)	14(17.1)	0.216	0.642
Yes	77(80.2)	68(82.9)		
Killip grade				
1	46(47.9)	9(10.7)	35.467	<0.001
2	10(10.4)	30(35.7)		
3	28(29.2)	27(32.1)		
4	12(12.5)	18(21.4)		
Atrial fibrillation				
No	91(94.8)	78(95.1)		>0.999
Yes	5(5.2)	4(4.9)		
Malignant ventricular arrhythmia				
No	87(90.6)	74(90.2)	0.007	0.931
Yes	9(9.4)	8(9.8)		

*Coronary angiography data*				
Number of diseased coronary vessels (except for LAD)				
1	62(64.6)	49(59.8)	0.501	0.778
2	27(28.1)	27(32.9)		
3	7(7.3)	6(7.3)		
SYNTAX score	19.21 ± 6.13	19.48 ± 6.14	-0.29	0.772
Collateral circulation				
0-Level	87(90.6)	74(90.2)	0.007	0.931
1-Level	9(9.4)	8(9.8)		

*Blood test*				
Uric acid	321.29 ± 57.80	329.05 ± 61.37	−0.867	0.387
Glycosylated hemoglobin	4.60 ± 0.92	6.04 ± 0.89	−10.599	<0.001
Low-density lipoprotein	2.97 ± 0.67	3.03 ± 0.74	−0.642	0.522
High-density lipoprotein	1.28 ± 0.27	1.26 ± 0.30	0.343	0.732
Creatinine	98.40 ± 37.45	98.00 ± 37.22	0.071	0.943
Glutamic-pyruvic transaminase	43.05 ± 16.55	45.33 ± 16.24	−0.925	0.356
FDP	3.05 ± 0.70	2.99 ± 0.65	0.589	0.556
Troponin I	24.72 ± 22.31	26.82 ± 14.82	−0.727	0.468
BNP	219.80 ± 106.78	267.30 ± 108.54	−2.936	0.004
NLR neutrophils/lymphocytes	6.45 ± 3.75	6.43 ± 2.56	0.048	0.961
Count of platelets	193.02 ± 33.61	196.93 ± 37.33	−0.734	0.464

Values are mean ± SD or *n* (%). BMI, body mass index; D2W, time from entrance to smooth passage of occluded blood vessel with a guidewire; ACEI/ARB, angiotensin-converting enzyme inhibitors/Angiotensin II receptor blockers; FDP, fibrinogen; BNP, brain natriuretic peptide; NLR, neutrophil/lymphocyte.

**Table 2:** Comparison of LVEDV and LVEF at baseline and after 6 months between the two groups of patients.

	Group	Baseline	6 months	Difference	*U*	*P*
LVEDV	Control group (*n* = 96)	53.05 ± 3.54	53.81 ± 7.38	0.76 ± 5.08	2880.50	<0.001
	Dapagliflozin group (*n* = 82)	54.00 ± 8.46	51.85 ± 8.38	−1.15 ± 2.65		

LVEF	Control group (*n* = 96)	45.33 ± 6.98	51.10 ± 9.10	5.77 ± 3.69	1061.50	<0.001
	Dapagliflozin group (*n* = 82)	39.24 ± 10.63	51.00 ± 10.12	11.76 ± 6.18		

Values are mean ± SD. LVEF, left ventricular ejection function; LVEDV, left ventricular end-diastolic volume.

**Table 3:** Comparison of clinical outcomes between the two groups of patients.

Variable	Control group *n* = 96	Dapagliflozin group *n* = 82	*t/χ* ^2^	*P*
Ventricular remodeling				
No	64 (66.7)	66 (80.5)	4.290	0.038
Yes	32 (33.3)	16 (19.5)		

**Table 4:** Single-factor logistics regression of ventricular remodeling.

Variable	B	Standard error	Wald	Degree of freedom	*P*	Exp(B)	95% confidence interval of EXP (B)	
							Lower limit	Upper limit
Dapagliflozin	−6.353	2.343	7.350	1	0.007	0.821	0.614	0.863
LVEDV	−0.218	0.117	3.462	1	0.063	0.804	0.639	1.012
LVEF	−0.513	0.177	8.388	1	0.004	0.598	0.423	0.847
BNP	−0.001	0.005	0.041	1	0.039	1.159	1.025	1.239
NLR	0.047	0.201	0.055	1	0.015	1.148	1.006	1.355
CnTI	0.217	0.073	8.769	1	0.003	1.243	1.076	1.435
Uric acid	0.014	0.010	2.068	1	0.150	1.014	0.995	1.034
Hb1AC	0.763	0.662	1.330	1	0.249	2.145	0.586	7.846
Diabetes history	0.722	1.227	0.346	1	0.556	2.058	0.186	22.796
ACEI/ARB	−6.687	2.356	8.053	1	0.005	0.723	0.457	0.851
*β*-block	−4.913	2.187	5.044	1	0.025	0.752	0.652	0.836
Constant	26.824	12.212	4.824	1	0.028	>1000		

**Table 5:** Multifactor logistics regression of dapagliflozin affecting ventricular remodeling.

Item	Confounding factors not adjusted		Confounding factors adjusted	
	*OR*(95%*CI*)	*Value*	*OR*(95%*CI*)	*Value*
Dapagliflozin group				
Dapagliflozin not used	1.0	—	1.0	—
Dapagliflozin used	0.815(0.673,0.968)	0.040	0.877(0.790,0.953)	0.024

a: Adjustment variable: taking ACEI/ARB, taking *β*-block, admission ejection fraction, troponin I, BNP, and NLR.

**Table 6:** Multifactor analysis of the effect of combined use of three drugs on ventricular remodeling.

Item	Confounding factors not adjusted		Confounding factor adjusted	
	*OR*(95%*CI*)	*Value*	*OR*(95%*CI*)	*Value*
Combined use of three drugs				
Used	1.0	—	1.0	—
Used	0.692(0.593,0.783)	0.026	0.754(0.673,0.854)	0.021

a: adjustment variable, admission ejection fraction, troponin I, BNP, and NLR.

## Data Availability

The data used to support the findings of this study are available from the corresponding author upon request.
